The article "Review on the Effect of Exercise Training on Immune Function" was retracted in 2023. Reasons: unreliable results or conclusions; concerns about the data; concerns about the peer review; concerns about the citations.

# Review on the Effect of Exercise Training on Immune Function

**DOI:** 10.1155/2022/9933387

**Published:** 2022-07-30

**Authors:** Feijiao Du, Cuicui Wu

**Affiliations:** Physical Culture Institute, Guizhou Normal University, Guiyang 550001, China

## Abstract

Exercise training is not only a necessary means to improve the level of exercise, but also an important means to improve the body's immunity. Different time, intensity, items, and forms of exercise training have different effects on the body's immune function. As a double-edged sword to improve the body's immune function, exercise training is a different reaction mechanism of different immune cells after exercise training. This paper combined with foreign scholars' studies on the immune function of the body of literature from different exercise intensity, different time, different sports, different movement forms, and different external environment such as angle of view for athletes body's immune cells and humoral immunity summarized the various indexes such as combing, in order to help academia, medicine, and sports. It provides enlightenment to the contemporary public on how to participate in sports training more healthily.

## 1. Introduction

As for the well-known viruses, “smallpox,” “SARS,” and “novel coronavirus” in recent years, the stronger the immunity of the body, the lower the incidence rate of virus infection. Contemporarily, people pay more attention to improving the immunity of the body. As the main means to improve and enhance the body's immunity, exercise training can effectively resist the risk of virus infection. Combined with the needs of society and the public, this paper classifies and summarizes previous studies and summarizes the effects of sports training on immune cells and humoral immunity in different time, intensity, project, and special environment, in order to provide reference for academic, medical, and sports circles.

## 2. The Effects of the Intensity of Exercise Training and Different Exercise on Immune Cells

### 2.1. Function of Immune Cells

Lymphocytes play a central role in the immune process of the body, and they can also secrete a variety of cytokines which can not only act on the immune cells themselves but also act on the nervous system and endocrine system to complete the immune function [1]. Macrophages are the core components of early physiological response after bone injury and late bone remodeling. Monocytes and macrophages are considered to play an important role in skeletal muscle repair and remodeling, mainly because they can promote the potential of angiogenesis, the secretion of growth factors, and the clearance of tissue fragments [2]. Dendritic cells are important outposts of the immune system and are responsible for presenting antigens to T cells. Dendritic cells are at the forefront of maintaining intestinal integrity, and they are professional antigen-presenting cells, including various subsets which are resident cells or migratory cells in lymphoid and nonlymphoid organs [3]. NK cells are the core members of the innate immune system, and they have the functions of early recognition and elimination of virus infection and tumor cells. At the same time, they are also the bridge between innate immunity and acquired immunity [4]. Neutrophils are the largest number of white blood cells in the blood. They are an important part of the body's nonspecific immune function and directly participate in the first “defense line” of the body's immune system [5]. Hematopoietic stem cells are mainly stored in the hematopoietic microenvironment of bone marrow and are the original cells of all immune cells. They are mainly responsible for inputting normal hematopoietic stem cells into the body of patients. They can enhance human hematopoietic and immune functions and effectively alleviate malignant blood diseases, genetic diseases, severe immunodeficiency, and other diseases [6].

#### 2.1.1. Effects of Different Intensity of Exercise Training on Immune Cells

When different intensity stimulation is used in sports training, the number of immune cells and immune function of the body will change, including the monitoring, self-stabilization, and defense of immune cells. Similarly, exercise training for different events has a different impact on the immune response of immune cells.

High-intensity exercise training has an adverse effect on most epidemic cells, especially the damage of long-term high-intensity exercise training to cells is very obvious, while the effect of short-term high-intensity exercise training on NK cells is more obvious. Regular moderate intensity exercise training can improve the body's immunity. In addition, long-term nonexercise will inhibit the function of immune cells.

#### 2.1.2. Effect of High-Intensity Exercise Training on Immune Cells

Foreign scholars have found that the intensity of exercise training affects the oxidation/antioxidant balance of lymphocytes and neutrophils, but only high-intensity exercise training will induce lymphocyte oxidative damage, which will cause oxidative damage to indicators such as erythrocytes and lymphocytes, but will not cause oxidative damage to neutrophils [7], which may be due to the decrease of catalase and glutathione peroxidase activities in neutrophils, glutathione peroxidase activity in lymphocytes, and the myeloperoxidase in neutrophils and the increase of catalase protein level in neutrophils. Shaw et al. found that resting peripheral blood type 2 and regulatory T-cells produced the anti-inflammatory cytokines interleukin 4 and interleukin 10, respectively, during high-intensity exercise training [8]. In addition, decreased secretory immunoglobulin A in elite athletes after high-intensity training leads to the alteration of mucosal immunity, which impairs the athlete's intracellular defense against pathogens and increases the incidence and risk of symptoms of upper respiratory tract symptoms [9]. In addition, the ratios of granulocytes/lymphocytes and lymphocyte/monocyte were shown to be sensitive to changes of fatigue [10]. Therefore, it can be used as an indicator of the body's cellular immunity and to evaluate the physiological state of its training state.

#### 2.1.3. Effects of Long-Term High-Intensity Exercise Training on Immune Cells

Long-term high-intensity training affects the function of innate immune cells, reduces the ability of immune cells to cope with acute exercise, and increases the risk of infection [11]. Long-term high-intensity exercise can also damage the function of macrophages which result in a reduction in macrophages and a decrease in phagocytic ability. The authors found, although a large amount of amino acid supplementation after exercise training, the degree of damage to macrophages could not be improved [12]. And Shephard and Shek [13] believed that NK cells recovered within 24 hours under long-term exercise training, and long-term high -intensity training would have adverse effects on immune surveillance and health of the body. In addition, Iwasaki and Medzhitov believed that a single prolonged exercise would impair the functions of T cells, NK cells, and neutrophils, alter the balance of type I and type II cytokines, and attenuate the immune response to primary and recall antigens in vivo.

#### 2.1.4. Effects of Short-Term High-Intensity Exercise Training on Immune Cells

There is a positive correlation between exercise and NK cell count and cytotoxic activity, and a short exercise affects the number and function of NK cells, but it does not affect the cytotoxicity of NK cells. Millard et al. [14] believed that short-term high-intensity exercise training may increase the number of NK cells but can reduce the toxicity of the cells, probably because NK cells rapidly redistribute between blood and tissues after acute exercise which causes the preferential redeployment of NK cell subsets with a well-differentiated phenotype and enhances cytotoxicity against HLA-expressing target cells. While a single exercise session induces the increase of leukocytosis and redistribution of effector cells between the blood compartment and lymphoid and peripheral tissues, this response is mediated by the increase of hemodynamics and the release of catecholamines and glucocorticoid following activation of the sympathetic nervous system.

#### 2.1.5. Effects of Moderate-Intensity Exercise Training on Immune Cells

Simpson et al.'s research shows that the improvement of immunity is due to regular moderate-intensity exercise. And regular moderate-intensity exercise has been shown to benefit cardiovascular health and reduce overall disease mortality. Regular short-term up to 45 minutes of moderate-intensity exercise is beneficial for immune defense [15]. Moderate-intensity exercise attenuates muscle ring finger 1-mediated atrophy of limb and respiratory muscles and improves limb muscle force production in mice with acute lung injury. Modulation of systemic neutrophil chemokine responses was by exercise training to restrict neutrophil influx into alveolar space. And early activity therapy attenuates muscle wasting and limits ongoing alveolar neutropenia by modulating systemic neutrophil chemokines in lung-injured mice and humans [16].

#### 2.1.6. Effects of Inactivity on Immune Cells

Prolonged bed rest significantly affects immune cell populations and cytokine concentrations. During spaceflight and simulated weightlessness (bed rest), immune function is suppressed, the number of granulocytes, natural killer, T cells, hematopoietic stem cells, and CD45RA and CD25 expressing T cells is increased, and the number of monocytes is significantly decreased. Exercise has different effects on the concentration of lymphocytes and B cells, but only regular exercise can enhance the immune function of human body functions [17].

### 2.2. The Effect of Training in Different Sports on Immune Cells

The number of T lymphocytes does not change after intensive exercise training by professionally trained athletes in cycling events, but exercise training or competition in cycling events can cause an increase in the number of myeloid cells in B cells, dendritic cells, and neutrophils. The number of T lymphocytes does not change after intensive exercise training by professionally trained athletes in cycling events, but exercise training or competition in cycling events can cause myeloperoxidase in B cells, dendritic cells, and neutrophils. There was an increase in the number of cells. Compared with cyclists, the immune cells of professional distance runners are more adversely affected, but there is no difference between the risk of respiratory tract infection and innate immune cells after long-term adaptation. The changes of immune cells are different in professional and amateur distance runners during the competition. In addition, swimming and running have different effects on the body's T cells. In swimming, men and women have different effects on cells. It reduced cytotoxicity of NK cells in volleyball pregame training.

#### 2.2.1. Effects of Cycling Training on Immune Cells

After completing a 20-minute continuous cycle cycling race at 80% VO2max, B cells increased by an average of 60% during exercise, with the largest increase in immature cells, followed by memory cells, and then naive cells [18]. Similarly, total dendritic cells increased by 150% during 80% VO2max exercise, plasmacytoid dendritic cells mobilized to a greater extent than myeloid dendritic cells, and plasmacytoid dendritic cells were preferentially mobilized during exercise, and exercise enhances immune surveillance by preferentially mobilizing effector cells [18]. After the cycle stage of professional cycling, myeloperoxidase in neutrophils increased, hemolysis and lymphopenia caused by exercise were negatively correlated with cell markers of oxidative stress [19]. The amount of ITN-Y produced by stimulated T lymphocytes at rest did not change in endurance trained male cyclists after a 6-day intensive training period. In endurance-trained male cyclists, the amount of ITN-Y produced at rest by stimulated T lymphocytes did not change after the intensive training period at a 6-day intensive training period. Neither acute nor chronic exercise training resulted in changes in circulating percentage or interleukin (IL)-4(+) (type 2) T lymphocyte counts [20].

#### 2.2.2. The Effects of Marathon Training on Immune Cells

Well-trained long-distance runners had significantly more muscle damage compared to the cyclists, and 3 days of functional overuse may result in significantly more muscle damage, soreness, and inflammation responses in runners, but upper respiratory symptoms and the decrease in innate immune after exercise have no difference. Linear increases in white blood cells, monocytes, and lymphocytes prior to initiation in ultraendurance runners in a multiphase ultramarathon; they increase before phase 3 and decrease thereafter. There was a significant increase in granulocytes followed by a decline to baseline until stage 3. Hemoglobin and hematocrit showed linear decline and had no changes in red blood cells and platelets throughout the multiphase ultramarathon [21]. Amateur middle-distance runners had significantly lower lymphocyte and eosinophil values prior to the start of the half-marathon than prerun values, while for mean red blood cell volume, platelets, mean platelet volume, white blood cells, neutrophils, and monocytes significantly decreased and then increased [22]. But the lymphocytes have increased in ultraendurance marathon runners before the marathon, while the number of lymphocytes decreased before the amateur half-marathon runners.

#### 2.2.3. The Effects of Swimming Sports on Immune Cells

Increased numbers of T cells in the blood after strenuous running and decreased numbers of lymphopenia after swimming exercise and the accumulation of T cells in the lungs and Peyer's patches may enhance immune alertness in these compartments, which are the body's main defensive barrier [23]. Oxidative damage in neutrophils and induction of antioxidant defense in lymphocytes, both neutrophil and lymphocyte responses to exercise are slightly weaker in women than in men .

#### 2.2.4. The Effects of Volleyball Exercise Training on Immune Cells

A-month preseason retraining (5 hours a day, 6 days a week) in college volleyball players significantly increased counts of CD56bright NK and CD56dim T cells (a subset with lower cytotoxicity) and decreased overall NK cell cytotoxicity from pretraining to posttraining, but the interleukin-6, interferon-gamma, and tumor necrosis factor-alpha levels did not change, and extensive training reduces total NK cell cytotoxicity as well as lysis units per NK cell [24].

#### 2.2.5. The Effect of Training on Immune Cells of Chinese Traditional Lianqi Sports

The cytotoxicity of natural killer cells increased by 60% immediately after lianqi training and returned to the basic level within 2 hours after training. The number of natural killer cell subsets did not change after lianqi training, and lianqi training had acute effects on natural killer cell activity [25].

## 3. Effects of Exercise Training in Special Environment on Immune Cells

### 3.1. Effects of Exercise Training in Cold or Hot Conditions on Immune Cells

Two 45-minute runs at 75-80% VO2max in cold, hot and humid conditions, white blood cell, neutrophil, and basophil counts increased significantly after exercise in both environments and more noticeable in hot environments. The activity of antioxidant enzymes and carbonyl index in lymphocytes and neutrophils were significantly increased or decreased, respectively, in a high temperature environment, and the lymphocyte expressions of catalase, H, and superoxide dismutase increased in hot conditions only after exercise [26]. The numbers of leukocytosis significantly increased immediately after intense actual fire-fighting exercises and firefighting activities and persisted after recovery. Most notably, plasma levels of ACTH and cortisol significantly elevated, and the number and percentage of lymphocytes significantly decreased, but the cortisol level still remained elevation after 90 minutes of recovery [27]. Leukocytes, neutrophils, lymphocytes, monocytes, platelets, mean platelet volume, interleukins, and cardiac troponin increased after a day of heavy training [28]. Exercise with protective clothing exacerbates the body's heat storage when compared with that in high temperatures, and because exercise alters the immune response and produces psychological and environmental stress on firefighters. In addition, fire instructors exposed to fires are 10 times more than firefighters, and physiological stress is also many times higher and 16 times more likely to experience symptoms of ill health [29].

### 3.2. Effects of Exercise Training at High Altitude on Immune Cells of the Body

Athletes, military personnel, firefighters, climbers, and astronauts need to train in extreme environments such as heat, cold, and high-altitude microgravity. Physical exercise in hot and thermoneutral conditions increases circulating stress hormones, catecholamines, and cytokines, with a concomitant increase in circulating white blood cells [30]. CD3(+) T lymphocytes significantly reduced during acute and chronic exposure to high altitude, the decline in T cells was entirely due to the decrease in CD4(+) T cells, and B lymphocytes were not affected by high-altitude exposure; natural killer cells significantly increased during acute and chronic exposure to high altitude, and the numbers of NK cell increased, but NK cytotoxic activity was not affected by high-altitude exposure [31]. Only in high altitude, even moderate exercise training also can activate the potential cytotoxic function of circulating granulocytes, but vigorous physical exercise strongly inhibits this activation, which prevents inflammatory damage and also activates the potential toxic function of circulating granulocytes [32].

## 4. The Influence of Psychological Index Changes on Immune Cells

Loss of T lymphocytes can negatively impact emotional health and cognition [33], and in a psychoneuroimmunological perspective, the immune system plays a role in the link between exercise and emotional health [34]. Study suggests that acute aerobic exercise may promote subjective emotional recovery from subsequent stressors and enhance emotional flexibility [35]. Chronic stress (lasting weeks/months/years) can suppress/dysregulated immune function, but acute stress (lasting minutes to hours) can have immune-enhancing effects. Dhabharet [36] found that short-term stress enhances the transporting, maturation, and function of dendritic cells, neutrophils, macrophages, and lymphocytes, which have been shown to enhance innate and adaptive immunity; chronic stress induces chronic increases of proinflammatory factors and inhibits the number, transport, and function of immune protective cells to suppress innate and adaptive immune responses by altering type 1 and type 2 cytokine balance.

### 4.1. Effects of Exercise Training after Sleep Interruption on Immune Cells

Nocturnal sleep disruption was associated with increased concentrations of total lymphocytes and CD3 (-)/CD56 (+) NK cells, mobilizing cytotoxic lymphocyte subsets (NK cells (including CD8 (+) T cells) *γ δ* T cells) have a greater response to exercise after sleep interruption at night, and the enhancement is more obvious 1 hour after exercise, and short-term changes in sleep structure will “activate” the immune system and lead to a slight enhancement of lymphocyte transport by acute dynamic exercise [37]. People who sleep less than six hours at a night are four times more likely to be diagnosed with an upper respiratory infection, which prevent more training. Since sleep restriction is considered an essential element of military training, future studies should examine interventions to reduce all negative effects on immunity and host defense [38]. Moreover, sleep interruption at night and exercise training with sleep time less than 6 hours per night will have an adverse impact on the production of immune cells and affect the kinetic energy of immune cells.

### 4.2. Effects of Different Periods of Exercise Training on Immune Cells

Foreign scholars studied the effect of repeated exercise in a day on the number of circulating leukocytes and NK cell activity. The results showed that the counts of leukocytes and neutrophils increased significantly both in the morning and afternoon after the exercise training. The change of lymphocyte count after exercise in the afternoon was more obvious, and the activity of NK cells was also significantly higher than that in the morning, indicating the interaction between exercise and diurnal effect. Two endurance exercises in one day had a “superposition effect” on the total number of leukocytes and neutrophils but did not affect the change of NK cell activity [39]. The number of NK cells in high-intensity training participants increased significantly during training in the morning and afternoon, the number of NK cells in high-intensity training participants decreased in the morning, but it was still significantly higher than the baseline level at 60 and 90 minutes after training in the morning; in the afternoon, the number of NK cells in high-intensity training participants decreased below the baseline level at 60 and 90 minutes after training, and the change of NK activity was mainly affected by day and night [40].

### 4.3. Effects of Supplements on Immune Cells after Exercise Training

Lactococcus lactis is a unique lactic acid bacteria, which can activate the plasma cell like dendritic cells and it can reduce the incidence rate and symptoms of upper respiratory tract infection by supplementing Lactococcus lactis to activate dendritic cells and reduce the fatigue accumulation of athletes during continuous high-intensity exercise. In addition, the intake of plasma will not affect muscle damage [41]. Wang et al. believed that taking Zhenqi Fuzheng Capsule can inhibit the decline of athletes' immune function caused by high-intensity training and accelerate the recovery of the body's immune function. It is widely believed that supplementing carbon compounds during long-term exercise can weaken the body's immune and endocrine response, but carbohydrate supplements will not affect the decline of body immunity after long-term exercise [42].

## 5. Conclusion

Each cell has its own unique immune function and has different effects on the body. Carrying out its own tasks, individuals form a complex and diverse strong immune system to maintain our health. Whether the general public or athletes or firefighters, they need a strong immune system to cooperate organically. There are different intensities of exercise training, such as long time high-intensity exercise on innate immune cells, and the body is adverse impact on health; in the usual sports training to avoid the process of long duration and high-intensity exercise, moderate intensity and regular exercise training to improve the body's immune function has good effect compared with the other strength of sports training, and not for a long time to exercise the body's immune function will be suppressed. Different sports training such as marathon, swimming, volleyball, and cycling have different change mechanisms on the immune cells of the body. Chinese traditional qi training has a certain influence on the immune function of the body. In the exercise training under the special environment of cold, hot, and high altitude, the adverse effect of hot environment on body immunity is greater than that of cold environment. The changes of psychological indicators, the number, and function of immune cells are different after sleep interruption and different periods of exercise training. Supplements after exercise training have a positive effect on the body's immune function. Through the above use of literature and materials to sort out, in order to bring help to the academic, medical, and sports circles, to the contemporary public on how to participate in sports training in a healthier way.

## Data Availability

The experimental data used to support the findings of this study are available from the corresponding author upon request.
